# Contrast-enhanced ultrasound perfusion quantification of solid liver lesions: First intraoperative characterization of tumor microvascularization

**DOI:** 10.1177/13860291251375539

**Published:** 2025-09-18

**Authors:** Laura S Kupke, Paul Kupke, Nina Käser, Moritz K Brandenstein, Liang Zhang, Christian Stroszczynski, Ernst-Michael Jung

**Affiliations:** 1 Department of Radiology, University Hospital Regensburg, Regensburg, Germany; 2 Department of Surgery, University Hospital Regensburg, Regensburg, Germany

**Keywords:** ultrasound, contrast-enhanced ultrasound, CEUS, microvascularization, intraoperative ultrasound, solid liver lesions

## Abstract

**Aim:**

Aim of the study was to differentiate solid liver lesions according to their microvascularization. Therefore, we analyzed perfusion using time intensity curves (TIC) measured during contrast-enhanced intraoperative ultrasound (CE-IOUS).

**Material and Methods:**

Data of 40 patients who underwent hepatic surgery with the diagnosis of hepatocellular carcinoma (HCC), intrahepatic cholangiocarcinoma (CCC), or liver metastases (LM) were retrospectively collected. CE-IOUS was performed using a linear multifrequency T-probe connected to a high-resolution device. Digital Imaging and Communications in Medicine (DICOM) loops were recorded, and TIC were analyzed for time to peak (TTP) and area under the curve (AUC) in tumor center, margin and reference tissue.

**Results:**

Analyses of the tumor center revealed significant higher AUC in HCC lesions than in CCC (*p* = 0.0310). HCC patients also showed longer TTP in reference tissue compared to CCC (*p* = 0.0251). Within the HCC cohort, TTP was shorter at tumor margins compared to reference tissue (*p* = 0.0420). For LM, AUC measured at tumor margins was higher than in center and reference tissue (*p*_center-margin_ = 0.0266, *p*_margin-reference_ = 0.0064).

**Conclusion:**

TIC analysis of solid liver lesions during CE-IOUS revealed significant differences in their microvascularization, improving, intraoperative differentiation. Artificial intelligence tools may enhance IOUS in the future by standardization and motion compensation.

## Introduction

Solid liver lesions are a frequent finding during abdominal imaging. The differentiation in benign and malignant lesions and the exact definition of the tumor entity is crucial for adequate therapy.^1,2^ In the group of primary malignant liver tumors, hepatocellular carcinomas (HCC) represent approximately 80% and cholangiocarcinomas (CCC) as the second most liver carcinoma after HCC about 5% to 30%.^3^ In addition, the liver is a highly metastasis-permissive organ especially for gastrointestinal tumors.^4^ Therefore, liver metastases (LM) are even more frequent than primary liver tumors.^5^

The first assessment to determine the tumor entity often is performed with transabdominal contrast-enhanced ultrasound (CEUS) due to its wide availability and cost-effectiveness.^6^ Contrast-enhanced intraoperative ultrasound (CE-IOUS) in particular is an important tool for successful tumor resection due to its high accuracy in describing and grading liver lesions.^7,8^ Therefore, an intravenous ultrasound contrast agent (UCA) is applied that helps to differentiate tumor lesions by visualizing the microcirculation.^9^ The UCA used is a suspension containing gas microbubbles which are exhaled by the patient a few minutes after injection. The UCA has the ability to remain intravascular thus enabling dynamic imaging of a lesion with tumor vessels and its surrounding microvascularization.^10,11^ Time-intensity curves (TIC) describing the bolus transit of UCA in the region of interest (ROI) can then be used for quantification of tumor perfusion.^12^ As different tumor entities show distinctive contrast dynamics, they can be differentiated according to the amount of UCA flowing through the tumor. HCC lesions typically show hyperenhancing in the early contrast phase and washout in the late phase.^13,14^ CCC lesions rather show inhomogeneous enhancement during the early phase and hypoenhancement in the late phase.^14^ LM on the other hand show rim enhancement to diffuse hyperenhancement in the early phase and tend to have a rapid washout in the late phase.^13,14^

In this study, we analyzed the perfusion of malignant solid liver lesions using TIC measured during CE-IOUS to optimize the differentiation of tumor entities during surgery.

## Materials and methods

### Data collection

For this retrospective and independent study, data were collected on 40 patients who underwent hepatic surgery with the diagnosis of HCC, CCC or LM between 09/2022 and 04/2024. In all cases, the diagnosis was confirmed by histopathological analyses and TIC were measured during CE-IOUS. Patients’ treatment was managed according to local guidelines.

The study was approved by the ethics committee of the University of Regensburg (approval number 18-1137-104).

### Conduction of CE-IOUS

For all intraoperative examinations a high-resolution ultrasound device (LOGIQ E9, GE Healthcare, Chicago, IL) equipped with a linear multifrequency T-probe (6–9 MHz) was used. An experienced attending radiologist (DEGUM III) performed the CE-IOUS. The UCA used for CEUS was a stabilized aqueous suspension of microbubbles composed of sulpur hexafluoride (SonoVue^®^, Bracco, Italy) resulting in an increased backscatter of ultrasound. The dynamic microvascularization of lesions can be visualized up to capillary changes due to the small size of the microbubbles (2–10 µm) and the ability to remain intravascular. 2.4–4.8 ml of UCA were administered centrally to perform CEUS.

### TIC analysis

Digital Imaging and Communications in Medicine (DICOM) loops of CE-IOUS were recorded for a duration of 60 s after application of UCA. Using an integrated software, 8 ROI with 5 mm of diameter were placed in the tumor center, margin and reference tissue to determine the lesions microvascularization. In these locations, TIC were generated and time to peak (TTP) and area under the curve (AUC) were analyzed. The ROI placement was performed according to the hospital's standard: 2 in the tumor center, 4 at the margin, 2 in the reference tissue. Figure 1 shows an exemplary TIC analysis.

**Figure 1.** Exemplary time-intensity curve (TIC) with device integrated software, region of interest (ROI) placement in the tumor center (yellow, light blue), at the margin (red, green, orange, purple) and in the reference tissue (gray, dark blue).

### Statistical analysis

Statistical calculations of the acquired data were made using GraphPad Prism (version 10, GraphPad Software Inc., San Diego, CA, USA). After assessment of non-parametric data, contingent on paired or non-matching data, Wilcoxon test or Mann-Whitney test were conducted. Results are expressed as indicated in the respective figure legends. *p*-value < 0.05 was considered statistically significant.

## Results

### Patient collective

The patient collective consisted of 25 males and 15 females with a median age of 65.95 years (IQR 58.33–71.78). Distributed on the surgery-indicating diagnosis, the population consisted of 20 LM (50.0%), 11 HCC (27.5%) and 9 CCC lesions (22.5%). In 29 cases (72.5%), surgery was conducted as planned after CE-IOUS, whereas in 8 cases (20.0%) additional local ablative therapy was applied and in 3 cases (7.5%) surgery had to be stopped due to extended tumor spread assessed by CE-IOUS (Table 1). The medians of TTP and AUC of the respective tumor entities are also shown in Table 1.

**Table 1.** 

**Patient Demographics**	
Median Age (years) [IQR]	65.95 [58.33–71.78]
Sex Distribution ♂/♀	25/15
**Surgery-Indicating Diagnosis**	
Liver Metastases (LM), n (%)	20 (50.0)
Hepatocellular Carcinoma (HCC), n (%)	11 (27.5)
Cholangiocarcinoma (CCC), n (%)	9 (22.5)
**Course of surgery**	
Resection, n (%)	29 (72.5)
Resection with additional local ablative therapy, n (%)	8 (20.0)
Stop of surgery, n (%)	3 (7.5)
**Median TTP (sec) [IQR]** **Median AUC [IQR]**	
HCC center	17.53 [11.26–30.61] 609.98 [258.96–1056.77]
HCC margin	11.94 [6.09–16.96] 393.53 [246.75–1012.77]
HCC reference	24.59 [13.40–26.90] 425.19 [194.00–590.74]
CCC center	12.61 [9.94–20.49] 139.18 [26.25–508.02]
CCC margin	12.54 [6.63–18.03] 481.18 [107.93–770.99]
CCC reference	8.69 [6.23–15.34] 354.07 [133.16–664.64]
LM center	13.77 [10.10–19.36] 415.70 [178.50–718.43]
LM margin	11.37 [9.69–15.55] 602.60 [452.81–763.61]
LM reference	13.59 [9.74–37.38] 494.43 [259.42–562.21]

### TIC analyses within one tumor entity

Within the HCC cohort, TTP was shorter at the tumor margins compared to reference tissue (*p* = 0.0420, Figure 2(a)).

**Figure 2.** Time intensity curve (TIC) analyses within one tumor entity. (a) Time to peak (TTP) within hepatocellular carcinoma (HCC) cohort; (b) TTP within cholangiocarcinoma (CCC) cohort; (c) and (d) area under the curve (AUC) within liver metastases (LM) cohort. Statistical analysis: Wilcoxon test, Appearance: median with interquartile range (whiskers min to max).

Patients with CCC showed a tendency in longer TTP in the tumor center than in reference tissue (*p* = 0.0742, Figure 2(b)).

For LM, the AUC measured at the tumor margin was higher than in the center (*p* = 0.0266, Figure 2(c)) and the reference tissue (*p* = 0.0064, Figure 2(d)). TTP measured in the corresponding localizations showed no difference.

### TIC analyses comparing different tumor entities

Compared to CCC patients, HCC patients showed a longer TTP in reference tissue (*p *= 0.0251, Figure 3(a)). Corresponding tendency was obtained between LM and CCC (*p *= 0.0768, Figure 3(b)).

**Figure 3.** Time intensity curve (TIC) analyses comparing different tumor entities. (a) reference tissue of hepatocellular carcinoma (HCC) and cholangiocarcinoma (CCC) cohort; (b) reference tissue of CCC and liver metastases (LM) cohort; (c) tumor center of HCC and CCC cohort; (d) tumor center of CCC and LM cohort. Statistical analysis: Mann-Whitney test. Appearance: median with interquartile range (whiskers min to max).

Analyses of the tumor center revealed a significant higher AUC in HCC lesions than in CCC (*p *= 0.0310, Figure 3(c)). LM again showed the same tendency compared to CCC (*p *= 0.0551, Figure 3(d)).

A comparison of TTP and AUC at the tumor margins among the different cohorts did not reveal differences.

## Discussion

Microvascularization of malignant solid liver lesions is a well-researched topic. Several studies showed differences between HCC, CCC and LM. Whereas HCC lesions usually show early hypervascularization followed by washout in the late phase, CCC lesions tend to have an inhomogeneous early enhancement followed by hypoenhancement and LM show rim enhancement and a rapid washout in the late phase.^13,14^ In this study, we pursued a first approach in analyzing the lesions’ microvascularization during CE-IOUS.

We obtained significant shorter TTP at the tumor margin compared to reference tissue within the HCC group. This also stands in line with the results of Schaible et al..^15^ The results can be explained by the theory that there is neovascularization at the tumor margins of HCC lesions leading to early hypervascularization in this region.^16^ In addition, HCC mostly occur in patients with liver cirrhosis. The blood flow in this altered liver tissue is less than in healthy liver tissue among other things due to rarefied blood vessels explaining the longer TTP.^17^ This phenomenon also explains the longer TTP of reference tissue in HCC patients compared to the ones with CCC.

The analysis of LM yielded in high AUC at the margin, indicating hypervascularization. This stands in line with generally known contrast behavior of LM with rim enhancement in the early contrast phase.^13,14^

Within the CCC group, we identified a tendency of longer TTP in the tumor center compared to reference tissue possibly following tumor necrosis.^18^ Furthermore, a late contrast uptake during the venous phase is described for CCC, which can also explain the longer TTP.^19^ This also stands in line with the significant lower AUC in the center of CCC lesions compared to HCC.

However, in this study we recorded TIC for only 60 s. In particular, washout of solid liver lesions is known to happen in the portal venous or late phase starting after 30 to 45 s.^20^ One limitation of this study therefore is that the washout kinetics could not be evaluated completely. For final discussion of tumor entities, the lesions’ late washout after 3 up to 5 min should be evaluated in the future also by TIC analysis.^13,14^

A second limitation of this study is that we did not preselect the patient collective according to the condition of their liver tissue or if they already underwent chemotherapy. Both could influence the lesions’ vascularization leading to altered results.^21,22^

Ultrasound in general is a dynamic procedure and its quality is depending on multiple variables. One point is the reader's experience – in this study, all ultrasounds were performed by an experienced sonographer (DEGUM III). However, the surgeons who were responsible for guiding the ultrasound probe were varying between the surgeries, possibly leading to a loss of quality. Another important disturbance factor are motion artifacts.^23^ During surgery, the patients are under general anesthesia which already is a very standardized setting. However, in the future artificial intelligence (AI) can help reduce artifacts and increase image quality by compensating for the mentioned sources of error. This can lead to longer and more stable recordings. Several studies already showed promising results for the application of AI in ultrasound, including diagnosis, prediction, monitoring and image procession.^24–27^ In addition, it was reported that CE-IOUS provides valuable information regarding intraoperative decision-making and that benefits outweigh the additional effort.^7,8^ Intraoperative TIC analysis can further optimize these intraoperative processes to achieve better outcomes for patients.

## Conclusion

TIC analysis of solid liver lesions during CE-IOUS showed significant differences in their microvascularization, improving the differentiation of tumor entities during surgery. It therefore should become a crucial interdisciplinary tool in tumor assessment. AI could help to improve the handling of IOUS in the future by using standardized protocols and compensating for motion artifacts, allowing for longer and more stable recordings.
